The article "Mitigation of NaCl Stress by Arbuscular Mycorrhizal Fungi through the Modulation of Osmolytes, Antioxidants and Secondary Metabolites in Mustard (Brassica juncea L.) Plants" was retracted in 2016. Reasons: manipulated results; errors in the data; errors in the methods; unreliable results or conclusions.

# Mitigation of NaCl Stress by Arbuscular Mycorrhizal Fungi through the Modulation of Osmolytes, Antioxidants and Secondary Metabolites in Mustard (*Brassica juncea* L.) Plants

**DOI:** 10.3389/fpls.2016.00869

**Published:** 2016-07-04

**Authors:** Maryam Sarwat, Abeer Hashem, Mohammad A. Ahanger, Elsayed F. Abd_Allah, A. A. Alqarawi, Mohammed N. Alyemeni, Parvaiz Ahmad, Salih Gucel

**Affiliations:** ^1^Department of Pharmaceutical Biotechnology, Amity Institute of Pharmacy, Amity UniversityNoida, India; ^2^Mycology and Plant Disease Survey Department, Plant Pathology Research Institute, Agriculture Research CenterGiza, Egypt; ^3^Botany and Microbiology Department, College of Science, King Saud UniversityRiyadh, Saudi Arabia; ^4^Stress Physiology Laboratory, Department of Botany, Jiwaji UniversityGwalior, India; ^5^Plant Production Department, College of Food and Agricultural Sciences, King Saud UniversityRiyadh, Saudi Arabia; ^6^Department of Botany, Sri Pratap CollegeSrinagar, India; ^7^Centre for Environmental Research, Near East UniversityNicosia, Cyprus

**Keywords:** AMF, antioxidants, *Brassica juncea*, flavonoids, lipid peroxidation, NaCl stress, osmolytes, phytohormones

## Abstract

Present work was carried out to investigate the possible role of arbuscular mycorrhizal fungi (AMF) in mitigating salinity-induced alterations in *Brassica juncea* L. Exposure to NaCl stress altered the morphological, physio-biochemical attributes, antioxidant activity, secondary metabolites and phytohormones in the mustard seedlings. The growth and biomass yield, leaf water content, and total chlorophyll content were decreased with NaCl stress. However, AMF-inoculated plants exhibited enhanced shoot and root length, elevated relative water content, enhanced chlorophyll content, and ultimately biomass yield. Lipid peroxidation and proline content were increased by 54.53 and 63.47%, respectively with 200 mM NaCl concentration. Further increase in proline content and decrease in lipid peroxidation was observed in NaCl-treated plants inoculated with AMF. The antioxidants, superoxide dismutase, ascorbate peroxidase, glutathione reductase, and reduced glutathione were increased by 48.35, 54.86, 43.85, and 44.44%, respectively, with 200 mM NaCl concentration. Further increase in these antioxidants has been observed in AMF-colonized plants indicating the alleviating role of AMF to salinity stress through antioxidant modulation. The total phenol, flavonoids, and phytohormones increase with NaCl treatment. However, NaCl-treated plants colonized with AMF showed further increase in the above parameters except ABA, which was reduced with NaCl+AMF treatment over the plants treated with NaCl alone. Our results demonstrated that NaCl caused negative effect on *B. juncea* seedlings; however, colonization with AMF enhances the NaCl tolerance by reforming the physio-biochemical attributes, activities of antioxidant enzymes, and production of secondary metabolites and phytohormones.

The article "Mitigation of NaCl Stress by Arbuscular Mycorrhizal Fungi through the Modulation of Osmolytes, Antioxidants and Secondary Metabolites in Mustard (Brassica juncea L.) Plants" was retracted in 2016. Reasons: manipulated results; errors in the data; errors in the methods; unreliable results or conclusions.

## Introduction

Salinity is a serious environmental constrain affecting the growth and development of most of the crop plants through out the globe (Giri et al., 2003; Hameed et al., 2014). According to Wang et al. (2003) 50% of land will be lost by salinity before the end of 21st century. NaCl is responsible for both hyperionic and hyperosmotic stress in plants due to the accumulation of Na^+^ ions, which disturbs many cellular processes such as photosynthesis, respiration and also affects the plasma membrane function. Increased Na^+^ accumulation alters the basic structure of the soil and results in decreasing soil porosity, consequently reducing soil aeration and conductance of water (Porcel et al., 2012). Its accumulation also creates low water potential in the soil, so hampers the uptake of water and mineral nutrients (Porcel et al., 2012). Salinity leads to oxidative stress through overproduction of reactive oxygen species (ROS) including singlet oxygen (^1^O_2_), hydrogen peroxide (H_2_O_2_), superoxide ion (), and hydroxyl radical (OH^•^). These ROS interact with cellular constituents including lipids, proteins as well as nucleic acids and disturb their normal functioning (Ahmad et al., 2008, 2010a; Ahmad, 2010).

Plants are well equipped with several defense mechanisms that help in averting the salt-triggered alterations. Compatible osmolytes such as proline, glycine betaine, soluble sugars, and sugar alcohols have been reported to assist plants in the tolerance mechanisms against environmental extremes (Ahmad et al., 2011, 2014). Both enzymatic and non-enzymatic antioxidants are present in plant cells, which mediate the scavenging of ROS; thereby, impede their aggregation and hence provides protection against oxidative damage (Ahmad et al., 2010a, 2011). Enzymatic antioxidants include superoxide dismutase (SOD), catalase (CAT), ascorbate peroxidase (APX), and glutathione reductase (GR; (Apel and Hirt, 2004). The non-enzymatic antioxidants, ascorbic acid (AsA), tocopherols, phenols, and thiols in combination with other antioxidants and phytohormones could contribute to improved tolerance against NaCl stress (Ahmad et al., 2010a, 2015; Rasool et al., 2013; Hashem et al., 2015).

In natural ecosystems, many microorganisms such as bacteria and fungi are able to colonize the roots of almost all plant species. Arbuscular mycorrhizal fungi (AMF) are ubiquitous as compared to other organisms inhibiting the rhizosphere. AMF enhances the plant growth and development by helping plants in the nutrient uptake and improving the rhizospheric soil health (Linderman, 1994; Al-Khaliel, 2010). AMF improves several physiological processes in host plants including water absorption potential of plants by increasing the hydraulic conductivity of roots (Al-Karaki and Clark, 1998; Ruiz-Lozano and Azcon, 2000; Ruiz-Lozano, 2003). These changes improved the growth of plants and subsequently recede the toxic ionic effect induced by salinity (Juniper and Abbott, 1993). The positive role of AMF in mitigating NaCl stress is also reported by Hashem et al. (2016) in *Ocimum basilicum* and Balliu et al. (2015) in *Solanum lycopersicum*. Symbiotic association of AMF with plants opens new alternatives for pyramiding strategies against salt stress (Dodd and Perez-Alfocea, 2012). To develop salt-tolerant plants is the greatest challenge in front of the scientific community, though little success has been achieved (Flowers, 2004; Munns and Tester, 2008; Schubert et al., 2009). It is assumed that the use of AMF could be a cost effective and sustainable approach to enhance the salt tolerance of economically important crops such as Indian mustard (*Brassica juncea* L.).

The article "Mitigation of NaCl Stress by Arbuscular Mycorrhizal Fungi through the Modulation of Osmolytes, Antioxidants and Secondary Metabolites in Mustard (Brassica juncea L.) Plants" was retracted in 2016. Reasons: manipulated results; errors in the data; errors in the methods; unreliable results or conclusions.

*B. juncea*, belongs to the family Brassicaceae, is an important oil-yielding crop throughout the globe. The production of edible oil in India is insufficient to fulfill the daily requirements. On the other hand, NaCl stress imposes adverse effects on growth and crop production of mustard plants. Therefore, the present study was aimed to investigate the (i) impact of NaCl stress on growth and metabolism of *B. juncea*, (ii) role of AMF in mitigating NaCl stress by modulating the biochemical attributes and antioxidants (enzymatic and non-enzymatic) and (iii) regulation of secondary metabolites and phytohormones by AMF in conferring tolerance against NaCl stress.

## Materials and Methods

### Mycorrhizal Inoculums

The tomato plants used as host were inoculated singly with AM fungi (*Glomus mosseae*; *G. fasciculatum*, and *G. macrocarpum*) for fungal spore propagation in green house with day/night temperature of 250°C/180°C, relative humidity 65%. The Hoagland’s solution without phosphorous was given to the plants for improved mycorrhizal colonization. The fungal spores were extricated from the trap culture and were estimated by the most probable number method (Alexander, 1982). The inoculum collected was composed of fungal spores, hyphae, and root fragments and was supplemented to the soil as 10 g of trap soil culture (approx. 100 spores per gram trap soil, *M* = 80%)/pot (1 kg). The soil without inoculum served as the reference.

The article "Mitigation of NaCl Stress by Arbuscular Mycorrhizal Fungi through the Modulation of Osmolytes, Antioxidants and Secondary Metabolites in Mustard (Brassica juncea L.) Plants" was retracted in 2016. Reasons: manipulated results; errors in the data; errors in the methods; unreliable results or conclusions.

### Pot Experiment

Certified seeds of *B. juncea* were treated with sodium hypochlorite (0.5%, v/v) for 5 min and then washed with distilled water and were allowed to germinate in growth chamber. The seedlings were transferred to pots (one seedling per pot) after germination and grown in a greenhouse for additional 3 weeks at an average day/night temperature 28°C/15°C. The composition of autoclaved experimental soil was 74.3% sand, 4.23% moisture, 0.17% carbon, 0.007% nitrogen, and 7.12 dS m^-1^ electrical conductivity (EC). Twenty-five-day-old plants with and without AMF were treated with different concentration of NaCl (0, 100, and 200 mM) dissolved in nutrient solution after every alternate day and the control was supplied with nutrient solution only. Each pot was supplemented with 100 ml of Hoagland’s solution to keep the soil moist. After 40 days of treatment (65-day-old plants at flowering stage), plants were harvested and analyzed for growth and biomass yield. Fresh leaf samples (fully expanded youngest leaf from top) were used to estimate the biochemical parameters and enzyme activities.

### Estimation of Growth Parameters

Length of the shoot and root was measured manually; however, for dry weight (DW) samples were dried in oven at 75°C for 72 h and then weighted.

### Estimation of Total Chlorophyll, Leaf Relative Water Content and Proline Content

Total chlorophyll in leaves was estimated by the method of Hiscox and Israelstam (1979). The absorbance was measured at 645 and 663 nm spectrophotometerically with DMSO as the reference.

The method of Smart and Bingham (1974) was used in the estimation of leaf relative water content (LRWC) and was calculated by the following equation:

LRWC(%) =FW−DW/TW−DW

For the proline estimation in leaves the method of Bates et al. (1973) was followed and the optical density (OD) was taken at 520 nm spectrophotometerically with toulene as the blank.

### Estimation of Hydrogen Peroxide (H_2_O_2_) and Lipid Peroxidation (MDA)

Hydrogen peroxide in leaves was determined according to the method of Velikova et al. (2000). The protocol of Heath and Packer (1968) protocol was followed for the estimation of MDA content. The OD was taken at 532 nm by subtracting the value of OD at 600 nm for correction of unspecific turbidity. 1% thiobarbituric acid (TBA) in 20% trichloroaceticacid (TCA) served as the blank.

### Antioxidant Enzyme Assay

Fresh leaf samples (10 g) were crushed in 100 mM Tris–HCl (pH 7.5) consisting of dithiothreitol (DTT) 5 mM, magnesium chloride (MgCl_2_) 10 mM, ethylenediaminetetraacetic acid (EDTA) 1 mM, magnesium acetate 5mM, and polyvinylpyrrolidine (PVP) 1.5%. The supernatant collected after centrifugation of homogenate served as the source for determination of SOD (EC 1.15.1.1), CAT (EC 1.11.1.6), and GR (EC 1.6.4.2). Same homogenizing medium was added with 2.0 mM AsA and was used for the determination of APX (EC 1.11.1.11).

The article "Mitigation of NaCl Stress by Arbuscular Mycorrhizal Fungi through the Modulation of Osmolytes, Antioxidants and Secondary Metabolites in Mustard (Brassica juncea L.) Plants" was retracted in 2016. Reasons: manipulated results; errors in the data; errors in the methods; unreliable results or conclusions.

The superoxide dismutase activity was estimated through the photoreduction of nitroblue tetrazolium (Van Rossun et al., 1997). The absorbance was read at 560 nm. One unit of SOD is the quantity of protein declining 50% photoreduction of NBT and was shown as unit per mg protein. The method of Luck (1974) was used for the determination of catalase activity. Absorbance was read at 240 nm and unit per mg protein expresses the catalase activity. Activity of APX was estimated following the protocol of Nakano and Asada (1981). The absorbance was read at 290 nm and unit mg^-1^ protein expresses the APX activity. One unit of APX is the quantity of protein used to degrade 1.0 μmol of substrate min^-1^ at 25°C. For the assay of glutathione reductase activity, the procedure of Carlberg and Mannervik (1985) was followed. The OD was read at 340 nm and the activity was expressed as unit mg^-1^ protein.

### Estimation of Ascorbate (AsA) and Reduced Glutathione (GSH)

Fresh leaf samples (500 mg) were crushed in an extraction buffer, meta-phosphoric acid (5%) in the presence of EDTA 1 mM. The supernatant collected was used as source for the estimation of ascorbate and glutathione content.

The method of Huang et al. (2005) and Paradiso et al. (2008) was employed for the assay of ascorbate (AsA) and glutathione (GSH), respectively.

### Determination of Hydrolytic Enzymes

The method of Shewale and Sadana (1978), Pressey and Avants (1980), and Cuglielminetti et al. (1995) was used for the estimation of α-amylase, carboxymethyl cellulase and cellulase and invertase activity, respectively. The unit h^-1^ mg^-1^ protein expresses the enzyme activity. The protocol described by Anson (1938) was followed for the assay of proteinase activity.

For the estimation of acid and alkaline phosphatase activities the procedure of Gianinazzi-Pearson and Gianinazzi (1976) was employed. The OD was taken at 410 nm and the enzyme activity was expressed as μmol p-nitrophenol released min^-1^ mg^-1^ protein.

### Determination of Total Phenolics and Flavonoids

Folin–Ciocalteu reagent method was used for the determination of phenolics (Chun et al., 2003) and mg gallic acid equivalent (GAE) g^-1^ extract expresses the total phenolic content. The protocol of Zhishen et al. (1999) was followed for the estimation of flavonoid content. The OD was taken at 510 nm and mg catechin equivalent g^-1^ extract expresses the flavonoid content.

The article "Mitigation of NaCl Stress by Arbuscular Mycorrhizal Fungi through the Modulation of Osmolytes, Antioxidants and Secondary Metabolites in Mustard (Brassica juncea L.) Plants" was retracted in 2016. Reasons: manipulated results; errors in the data; errors in the methods; unreliable results or conclusions.

### Estimation of Phytohormones

The procedure described by Kusaba et al. (1998) was employed for the estimation of pytohormones [indole-3-acetic acid (IAA), indole-3-butyric acid (IBA), and abscisic acid (ABA)]. The leaf tissue (500 mg) was crushed in 80% aqueous acetone in the presence of 10 mg butylated hydroxytoluene. Ethyl acetate (EtOAc) and sodium bicarbonate (NaHCO_3_) were used to purify the homogenate. The purified sample was loaded in column of PEGASIL ODS (6 mm i.d. × 150 mm) for HPLC. For the blank, 10–200 ng ml^-1^ pure phytohormones was used.

### Statistical Analysis

One-way analysis of variance (ANOVA) was used followed by Duncans Multiple Range Test (DMRT) for the statistical analysis. The values obtained are mean ± SE for five replicates in each group. *P* values ≤ 0.05 were considered as significant.

## Results

### AMF Improved Growth and Biomass Yield in NaCl-Treated Mustard Plants

Salt stress caused reduction in growth in terms of height and dry weight (**Figures 1A–C**). Shoot length is decreased by 30.64 and 50.39% at 100 and 200 mM NaCl concentration, respectively in comparison to control. Treatment with AMF showed an increase by 30.92% at 100 mM+AMF and 30.36% at 200 mM+AMF in shoot length as compared to 100 and 200 mM NaCl treatment alone (**Figure 1A**). The maximum root length is decreased by 39.08% at 200 mM NaCl treatment over the control, but supplementation with AMF showed only 30% decrease in the root length at 200 mM+AMF treatment (**Figure 1B**). Increase in NaCl concentration causes a decrease in shoot dry weight (DW) by 50.26% at 200 mM NaCl concentration relative to control. Application of AMF showed an increase by 31.30% in DW at 200 mM+AMF treatment over NaCl-treated plants alone (**Figure 1C**).

**FIGURE 1:** **Effect of different concentrations of NaCl in the presence and absence of AMF on **(A)** Shoot length, **(B)** root length, and **(C)** shoot dry weight in *Brassica juncea* L.** Data presented are the mean ± SE (*n* = 5). Different letters indicate significant differences among treatments at *P* ≤ 0.05 level.

### AMF Enhanced Total Chlorophyll, Relative Water Content and Proline Content in Mustard Plants Subjected to NaCl Stress

The results pertaining to the impact of NaCl and AMF on total chlorophyll, relative water content (RWC), and proline content are depicted in **Figures 2A–C.** NaCl concentration of 200 mM caused a decrease in total chlorophyll content by 40.08%; however, addition of AMF to plants treated with NaCl showed enhancement in the chlorophyll content by 28.48 and 27.46% at 100 mM+AMF and 200 mM+AMF treatments, respectively in comparison to NaCl-treated plants alone (**Figure 2A**).

The article "Mitigation of NaCl Stress by Arbuscular Mycorrhizal Fungi through the Modulation of Osmolytes, Antioxidants and Secondary Metabolites in Mustard (Brassica juncea L.) Plants" was retracted in 2016. Reasons: manipulated results; errors in the data; errors in the methods; unreliable results or conclusions.

**FIGURE 2:** **Effect of different concentrations of NaCl in the presence and absence of AMF on **(A)** total chlorophyll, **(B)** leaf water content, and **(C)** proline content in *Brassica juncea* L.** Data presented are the mean ± SE (*n* = 5). Different letters indicate significant differences among treatments at *P* ≤ 0.05 level.

A decrease of 31.82 and 45.05% in RWC was observed at 100 and 200 mM NaCl concentration, respectively, relative to control. Co-inoculation of AMF restored the RWC and showed an increase of 37.21% at 100 mM+AMF and 35.32% at 200 mM+AMF treatments over NaCl-treated plants (**Figure 2B**).

Application of NaCl caused an elevation in the proline content by 2.03-fold and 4.53-fold with 100 and 200 mM treatments, respectively relative to control. Application of AMF further enhanced the proline content by 1.72-fold at 100 mM+AMF and 1.65-fold at 200 mM+AMF over the plants treated with NaCl alone (**Figure 2C**).

### AMF Reduces the H_2_O_2_ Accumulation and Lipid Peroxidation in NaCl-treated Mustard Plants

The effect of AMF on H_2_O_2_ level and membrane lipid peroxidation in mustard seedlings suffering from salt stress is shown in **Figures 3A,B.** H_2_O_2_ is increased by 1.99-fold and 3.35-fold at 100 and 200 mM NaCl concentration, respectively over the control. Co-application of AMF with NaCl declines the accumulation of H_2_O_2_ by 1.24-fold at 100 mM+AMF and 2.36-fold at 200 mM+AMF relative to control.

**FIGURE 3:** **Effect of different concentrations of NaCl in the presence and absence of AMF on **(A)** H_2_O_2_, and **(B)** malondialdehyde (MDA) content in *Brassica juncea* L.** Data presented are the mean ± SE (*n* = 5). Different letters indicate significant differences among treatments at *P* ≤ 0.05 level.

Lipid peroxidation, measured as malondialdehyde (MDA) content, is increased exponentially in NaCl-treated plants with a maximum accumulation of 2.19-fold at 200 mM (**Figure 3B**). However, AMF-inoculated plants showed a decline in the MDA content by 1.17-fold and 1.72-fold at 100 mM+AMF and 200 mM+AMF treatments, respectively over control plants.

### AMF Enhanced the Activity of Enzymatic Antioxidants in Mustard Seedlings Treated with NaCl

The results related to the effect of NaCl and AMF on enzymatic antioxidants are depicted in **Figures 4A–D.** SOD activity is increased by 64.29 and 93.63% at 100 and 200 mM NaCl treatments, respectively relative to control. Application of AMF in the presence of NaCl further increases the SOD activity by 47.14% at 100 mM+AMF and 37.57% at 100 mM+AMF treatments over NaCl-treated plants alone (**Figure 4A**).

**FIGURE 4:** **Effect of different concentrations of NaCl in the presence and absence of AMF on activities of **(A)** superoxide dismutase (SOD), **(B)** catalase (CAT), **(C)** ascorbate peroxidase (APX), and **(D)** glutathione reductase (GR) in *Brassica juncea* L.** Data presented are the mean ± SE (*n* = 5). Different letters indicate significant differences among treatments at *P* ≤ 0.05 level.

The article "Mitigation of NaCl Stress by Arbuscular Mycorrhizal Fungi through the Modulation of Osmolytes, Antioxidants and Secondary Metabolites in Mustard (Brassica juncea L.) Plants" was retracted in 2016. Reasons: manipulated results; errors in the data; errors in the methods; unreliable results or conclusions.

CAT activity is decreased by NaCl treatment, however application of AMF enhanced the CAT activity by 45.92 and 27.50% at 100 mM+AMF and 200 mM+AMF treatments, respectively over the plants treated with NaCl alone (**Figure 4B**).

The APX activity is increased by 58.30% at 100 and 121.54% at 200 mM NaCl treatments over the control. Co-inoculation of AMF further increases the APX activity by 31.96 and 14.89% at 100 mM+AMF and 200 mM+AMF treatments, respectively comparison to NaCl-treated plants (**Figure 4C**).

GR activity is also increased with increasing NaCl concentrations. Maximum increase of 43.85% is recorded at 200 mM NaCl treatment as compared to control. Salt-treated plants supplemented with AMF showed further increase of 21.92% in GR activity at 200 mM+AMF treatment as compared to NaCl-treated plants (**Figure 4D**).

### AMF Improved the Non-enzymatic Antioxidants in NaCl-Treated Mustard Plants

Increasing NaCl concentrations caused a decrease in AsA content by 35.41% at 100 and 50.00% at 200 mM treatments as compared to control. However, AMF-inoculated plants showed increase of 12.90 and 18.75% at 100 mM+AMF and 200 mM+AMF treatments, respectively relative to plants treated with NaCl alone (**Figure 5A**).

**FIGURE 5:** **Effect of different concentrations of NaCl in the presence and absence of AMF on contents of **(A)** ascorbic acid (AsA) and **(B)** glutathione (GSH) in *Brassica juncea* L.** Data presented are the mean ± SE (*n* = 5). Different letters indicate significant differences among treatments at *P* ≤ 0.05 level.

Glutathione is increased by 44.00% at 100 and 80.00% at 200 mM NaCl treatments in comparison to control. Inoculation of NaCl-treated plants with AMF further increased the glutathione content by 19.44 and 17.77% at 100 mM+AMF and 200 mM+AMF treatments, respectively over the plants treated with NaCl alone (**Figure 5B**).

### AMF Maintains the Activities of Hydrolytic Enzymes in Mustard Plants under NaCl Stress

The effect of NaCl and AMF on hydrolytic enzyme activities is depicted in **Table 1.** NaCl concentration (200 mM) enhanced the carboxymethyl cellulase (CMCase), cellulase, invertase, and protease activity by 67.84, 55.98, 61.03, and 61.95%, respectively relative to control, however, inoculation with AMF to NaCl-treated plants showed a decline by 12.88% in CMCase, 25.90% in cellulase, 16.12% in invertase, and 28.85% in protease activity at 200 mM+AMF treatment over NaCl-treated plants alone. NaCl decreases the amylase activity and maximum decrease by 43.32% was observed at 200 mM NaCl treatment. Co-inoculation of AMF showed a further decrease of 18.53% in amylase activity at 200 mM+AMF treatment over plants treated with NaCl (**Table 1**).

The article "Mitigation of NaCl Stress by Arbuscular Mycorrhizal Fungi through the Modulation of Osmolytes, Antioxidants and Secondary Metabolites in Mustard (Brassica juncea L.) Plants" was retracted in 2016. Reasons: manipulated results; errors in the data; errors in the methods; unreliable results or conclusions.

**Table 1:** Effects of AMF on hydrolytic enzyme activity of mustard plants under salt stress.

Treatments	Hydrolytic enzyme activity (EU mg^-1^ protein)				
	
	Amylase	CMCase	Cellulase	Invertase	Protease
0 mM	4.57 ± 0.61a	21.55 ± 1.24e	4.43 ± 0.62e	2.31 ± 0.24e	2.76 ± 0.31d
0+AMF	3.92 ± 0.49b	18.41 ± 1.12f	4.02 ± 0.58e	2.01 ± 0.18e	2.33 ± 0.25f
100 mM	3.81 ± 0.41c	29.32 ± 1.37c	5.52 ± 0.78b	2.98 ± 0.34c	3.55 ± 0.48b
100 mM+AMF	3.01 ± 0.35d	23.12 ± 1.28d	4.73 ± 0.69d	2.39 ± 0.27d	2.72 ± 0.28de
200 mM	2.59 ± 0.27e	36.17 ± 1.81a	6.91 ± 0.85a	3.72 ± 0.51a	4.47 ± 0.67a
200 mM+AMF	2.11 ± 0.19f	31.51 ± 1.64b	5.12 ± 0.74bc	3.12 ± 0.40b	3.18 ± 0.41c


*Data presented are the mean ± SE (*n* = 5). Different letters next to the number indicate significant difference (*P* < 0.05).*

*FW, fresh weight; DW, dry weight.*

### AMF Enhances the Acid and Alkaline Phosphatase Activities in Mustard Plants under NaCl Stress

The results related to the effect of NaCl and AMF on acid and alkaline phosphatase activities is depicted in **Figures 6A,B.** NaCl stress increases the acid phosphatase activity by 105.90 and 259.09% at 100 and 200 mM NaCl concentration, respectively as compared to control. Further enhancement is observed with the application of AMF to NaCl-treated plants (**Figure 6A**).

**FIGURE 6:** **Effect of different concentrations of NaCl in the presence and absence of AMF on **(A)** acid phosphatase and **(B)** alkaline phosphatase in *Brassica juncea* L.** Data presented are the mean ± SE (*n* = 5). Different letters indicate significant differences among treatments at *P* ≤ 0.05 level.

Maximum increase of 259.40% was recorded in alkaline phosphatase activity with 200 mM NaCl concentration over control. Further increase of 8.81% was recorded in plants under 200 mM+AMF treatment as compared to plants treated with 200 mM NaCl (**Figure 6B**).

### AMF Improved the Total Phenolics, Flavonoids, and Phytohormones in Mustard Plants under NaCl Stress

Total phenol content is increased with increasing NaCl concentrations reaching a maximum of 192.80% at 200 mM NaCl treatment over the control. NaCl-treated plants inoculated with AMF (200 mM+AMF) showed further increase of 60.93% in total phenol content relative to plants treated with NaCl (**Table 2**).

The article "Mitigation of NaCl Stress by Arbuscular Mycorrhizal Fungi through the Modulation of Osmolytes, Antioxidants and Secondary Metabolites in Mustard (Brassica juncea L.) Plants" was retracted in 2016. Reasons: manipulated results; errors in the data; errors in the methods; unreliable results or conclusions.

**Table 2:** Effects of AMF on total phenol, flavonoid, IAA, IBA, and ABA parameters of mustard plants under salt stress.

Treatments	Total phenol (mg GAE g^-1^ extract)	Flavonoid (mg catechin g^-1^ extract)	IAA (mmol g^-1^ FW)	IBA (mmol g^-1^ FW)	ABA (mmol g^-1^ FW)
0 mM	4.31 ± 0.59f	14.51 ± 1.21f	1.32 ± 0.07d	88.32 ± 2.67c	0.73 ± 0.02e
0+AMF	8.47 ± 0.88d	15.32 ± 1.29e	2.71 ± 0.29a	141.22 ± 4.98a	0.49 ± 0.008f
100 mM	7.11 ± 0.69e	19.87 ± 1.47d	0.95 ± 0.03e	62.75 ± 1.78e	3.55 ± 0.44c
100 mM+AMF	13.22 ± 1.1b	22.74 ± 1.63c	2.02 ± 0.18b	103.70 ± 3.55b	1.91 ± 0.14d
200 mM	12.62 ± 1.00c	24.53 ± 1.77b	0.72 ± 0.01f	47.18 ± 1.49f	6.87 ± 0.83a
200 mM+AMF	20.31 ± 1.47a	27.91 ± 1.89a	1.71 ± 0.12c	79.13 ± 2.34d	3.72 ± 0.54b


*Data presented are the mean ± SE (*n* = 5). Different letters next to the number indicate significant difference (*P* < 0.05).*

*FW, fresh weight; DW, dry weight.*

The flavonoid content is increased by 36.94 and 69.05% at 100 and 200 mM NaCl treatments over control. However, plants treated with AMF showed further increase in flavonoid content by 14.44 and 13.77% at 100 mM+AMF and 200 mM+AMF treatments, respectively as compared to NaCl-treated plants (**Table 2**).

NaCl stress decreases IAA and IBA and the maximum decrease of 45.45% in IAA and 46.58% in IBA was observed at 200 mM NaCl relative to control (**Table 2**). Plants supplemented with AMF showed increase of 137.50% and 67.71% in IAA and IBA, respectively as compared to 200 mM NaCl-treated plants (**Table 2**). NaCl stress caused an increase in ABA content by 386.30% at 100 mM and 841.09% at 200 mM NaCl treatments compared to control. Addition of AMF decreases the ABA concentration by 46.19 and 45.85% at 100 mM+AMF and 200 mM+AMF, respectively in comparison to NaCl-treated plants (**Table 2**).

## Discussion

### AMF Improved Growth and Biomass Yield in NaCl-Treated Mustard Plants

Plant growth and biomass are severely reduced under salt stress, might be due to the non-availability of nutrients. Our study with *Brassica* showed improved growth and biomass in AMF-inoculated plants. Other reports (Al-Karaki, 2000; Giri et al., 2003; Hashem et al., 2014) also showed better growth in AMF-inoculated plants in comparison to non-inoculated plants under salt stress. Increased root and shoot dry weight is observed in mycorrhizal than the non-mycorrhizal seedlings of *Acacia nilotica* (Giri et al., 2007), tomato (Al-Karaki, 2000), and *Cucurbita pepo* (Colla et al., 2008). It has been proposed that increased growth and biomass in AMF-colonized plant might be due to enhanced nutrient acquisition, especially better P nutrition through the mycorrhizae (Evelin et al., 2009). Kohler et al. (2009) showed enhanced uptake of essential mineral elements in lettuce plants subjected to severe salt stress inoculated with AMF compared to the uninoculated plants.

The article "Mitigation of NaCl Stress by Arbuscular Mycorrhizal Fungi through the Modulation of Osmolytes, Antioxidants and Secondary Metabolites in Mustard (Brassica juncea L.) Plants" was retracted in 2016. Reasons: manipulated results; errors in the data; errors in the methods; unreliable results or conclusions.

### AMF Enhanced Total Chlorophyll, Leaf Relative Water Content, and Proline Content

Our results of reduced chlorophyll content under NaCl stress corroborate with the reports of Doganlar et al. (2010), Rasool et al. (2013), and Alqarawi et al. (2014) for *Lycopersicon esculentum*, *Cicer arietinum*, and *Ephedra alata*, respectively. This reduction can be attributed to the enhanced chlorophyllase activity which causes pigment degeneration. These degraded pigments cause reduction in photosynthesis and hence the growth is affected. Reports are available on negative effect of salinity on protein synthesis and protein-pigment complex functioning (Levitt, 1980; Sultana et al., 1999; El-Tayeb, 2005). In comparison to the salt-stressed plants, the AMF-inoculated plants have enhanced chlorophyll contents. These results are in synergy with the findings of Hajiboland et al. (2012) on *Solanum lycopersicum* L. and Aroca et al. (2013) on *Lactuca sativa*. The higher chlorophyll content causes increased photosynthesis and thus increased growth. While analyzing the mechanism behind increased chlorophyll content in AMF colonized plant, it was shown by Sheng et al. (2008) that enhanced mineral uptake especially magnesium could be one of the reasons.

The increased plant growth exhibited by AMF-inoculated plant in our study can also be attributed to improved absorption of water by plant roots. Studies have shown enhancing root hydraulic conductivity, osmotic balance and composition of carbohydrates in AMF-colonized plants, which further contributes to increased water potential (Evelin et al., 2009). The increased water potential also dilutes the toxicity of the sodium ions (Juniper and Abbott, 1993).

NaCl stress causes increase in the proline content, this corroborates with the findings of Ahmad (2010), Azooz et al. (2011), and Rasool et al. (2012). The mechanism behind enhanced proline accumulation may be the increased activity of proline synthesizing enzymes or reduced catabolizing enzymes or both (Jaleel et al., 2007; Ahmad et al., 2010b). Mycorrhizal colonization further increases the proline accumulation under NaCl stress (Shekoofeh et al., 2012). Kumar et al. (2010) also reported an increased level of proline and soluble sugars in AMF-inoculated *Jatropha curcas* as compared to non-inoculated plants under salinity stress. AMF inoculation also increases the tolerance capacity of plants by stabilizing osmotic homeostasis and quenching toxic radicals (Feng et al., 2002; Ahmad et al., 2014).

The article "Mitigation of NaCl Stress by Arbuscular Mycorrhizal Fungi through the Modulation of Osmolytes, Antioxidants and Secondary Metabolites in Mustard (Brassica juncea L.) Plants" was retracted in 2016. Reasons: manipulated results; errors in the data; errors in the methods; unreliable results or conclusions.

### AMF Modulates the Accumulation of H_2_O_2_, MDA, and Antioxidants in Mustard Plants Treated with NaCl

Salt stress increases H_2_O_2_ production, which results in membrane leakage in mustard (Ahmad, 2010; Ahmad et al., 2012). Tuna et al. (2008) also confirms ROS-induced membrane leakage and disturbance in cellular homeostasis in salinity-stressed plants. AMF-treated plants showed increased activity of antioxidants, which might lead to reduced production of H_2_O_2_. Increased MDA content in the present study coincides with the reports of Rasool et al. (2013) in chickpea. NaCl-treated plants inoculated with AMF showed lower lipid peroxidation, which might be due to enhanced scavenging of ROS by antioxidants (Hashem et al., 2014, 2015). Qun et al. (2007) and Tang et al. (2009) suggested the role of AMF in increasing antioxidant activities and phosphate metabolism for the protection of membrane lipids.

Environmental stress cause increased activities of different antioxidant enzymes. These enzymes help in scavenging of toxic ROS and hence protecting the plant biomolecules from oxidative damage (Ahmad et al., 2015). We have found increased activities of SOD, APX, and GR in the present study and similar reports are there for *Sesamum indicum* (Koca et al., 2007), and *C. arietinum* (Rasool et al., 2013). SOD scavenges superoxide radicals to water and hydrogen peroxide, CAT and APX converts this H_2_O_2_ into water and oxygen. In our study, AMF-inoculated plants show further enhancement in the activity of antioxidant enzymes thus increasing the ROS scavenging capacity. Qun et al. (2007) and Abdel Latef and Chaoxing (2011) also reported that AMF-inoculated plants increased the activity of antioxidant enzymes in tomato under salt stress. Arbuscular mycorrhiza possesses various *SOD* genes, which get up-regulated and provides tolerance to the inoculated plants against oxidative damage (Wu et al., 2010; Hajiboland et al., 2012). AMF enhanced the expression of *SOD* gene under drought stress in *Poncirus trifoliata* resulting in lower accumulation of ROS in *Poncirus trifoliata* (Huang et al., 2014). *SOD* gene expression was also enhanced in lettuce plants inoculated with AMF under drought stress (Ruiz-Lozano et al., 2001). CAT decreased with elevated levels of NaCl and may be due to its lower affinity for scavenging H_2_O_2_ than APX. Both APX and CAT played an important role in the elimination of H_2_O_2_ under oxidative stress. Increased activity of antioxidant enzymes in AMF colonized plants are also accompanied with less accumulation of MDA content indicating the mitigation of oxidative burst by AMF. Plants inoculated with AMF improved the production of various antioxidative enzymes through the availability of metals to the enzymes such as CAT, POX, and SOD (Alguacil et al., 2003). Deficiencies and excesses of metals changed the expression of different metalloenzymes, e.g., Fe availability enhanced the activities of CAT and APX in *Nicotiana plumbaginifolia* (Kamfenkel et al., 1995). The availability of metals such as Fe, Cu, Zn, and Mn in plants inoculated wih AMF might be the reason of increased activity of SOD (Evelin et al., 2009).

The article "Mitigation of NaCl Stress by Arbuscular Mycorrhizal Fungi through the Modulation of Osmolytes, Antioxidants and Secondary Metabolites in Mustard (Brassica juncea L.) Plants" was retracted in 2016. Reasons: manipulated results; errors in the data; errors in the methods; unreliable results or conclusions.

In our study, we reported that NaCl declined the non-ezymatic antioxidants, *viz.*, AsA and glutathione. AsA has a key role in antioxidant network. Ascorbate has been reported to be involved in cell division, expansion of cell wall, and other developmental processes (Pignocchi and Foyer, 2003). AsA-GSH cycle has an essential role in plant resistance under stress conditions (Anjum et al., 2011). Glutathione detoxifies the excess of H_2_O_2_ and keeps ROS level under control (Rausch et al., 2007). H_2_O_2_ was detoxified by APX in to H_2_O using ascorbate (AsA) as the major substrate and GSH continuously restores ascorbate (AsA) from dehydroascorbate (DHA), through AsA-GSH cycle (Foyer et al., 1997). In this process, GSH is oxidized into GSSG, which is subsequently recycled by GR. Increase in glutathione content due to NaCl stress is in corroboration with Hasanuzzaman et al. (2014) who also reported increase in glutathione content in *Brassica napus* under salt stress. AsA pool signifies the involvement of AMF through the regeneration of AsA via increased GR activity and GSH availability (Anjum et al., 2010) (**Figure 7**). A higher activity of GR provides NADP^+^ to accept the electrons generated in the photosynthetic electron transport, thus decreasing the production of  (Menconi et al., 1995).

**FIGURE 7:** **Negative effects of NaCl stress and the mitigating role of AMF in plants**.

### AMF Regulates Hydrolytic Enzyme Activities in Mustard Plants under NaCl Stress

In the present study, decrease in α-amylase activity was observed with elevated NaCl concentration. Similar findings were reported by Sangeetha (2013) in *Zea mays* and Thakur and Sharma (2005) in *S. bicolor*. During stress, starch gets degraded, mainly due to the amylase activity (Thakur and Sharma, 2005). It has been reported that increase in sugar is accompanied by a decrease in starch content due to the activity of α-and β-amylases (Monerri et al., 1986; Gupta et al., 1993). NaCl decreased amylase activity that in turn reduced the transport of assimilates, so the growth and development of plant is affected (Hashem et al., 2015). The hydrolytic enzyme activities, i.e., CMCase, cellulase, invertase, and protease are increased with increasing concentration of NaCl in our results. Thakur and Sharma (2005) also reported increased invertase activity in *Sorghum* plants subjected to NaCl stress. Similarly, Kennedy and De Fillippis (1999) showed increased protease activity in *Grevillea* species under NaCl stress.

The article "Mitigation of NaCl Stress by Arbuscular Mycorrhizal Fungi through the Modulation of Osmolytes, Antioxidants and Secondary Metabolites in Mustard (Brassica juncea L.) Plants" was retracted in 2016. Reasons: manipulated results; errors in the data; errors in the methods; unreliable results or conclusions.

### AMF Enhances the Acid and Alkaline Phosphatase Activities in Mustard Plants under NaCl Stress

The acid and alkaline phosphatase activities are also increased with elevated NaCl levels in our study. Similar results were shown by Ehsanpour and Amini (2003) in *Medicago sativa* and Olmos and Hellin (1997) in *Pisum sativum* under NaCl stress. Stephen et al. (1994) demonstrated the deficient uptake of P in pea seedlings leads to decreased phosphatase activity. According to Pan and Chen (1988), there may be two reasons for higher activity of acid phosphatase: (i) high resistance of pre-existing acid phosphatase to stress-induced enzyme degradation and (ii) synthesis of new acid phosphatase due to stress. The increase in alkaline phosphatase by NaCl stress coincides with the finding of Rai and Sharma (2006) in *Anabaena doliolum*. AMF inoculated plants showed increase in α-amylase activity, might be due to the enhanced levels of IAA and other phytohormones (Kim et al., 2006). Sheng et al. (2008) reported that AMF-inoculated plants under NaCl stress try to maintain the hydrolytic enzyme activities for the normal growth and maintenance through restoration of water balance and higher stomatal conductance. This increases the water demand for transpiration. According to Evelin et al. (2009) AMF-treated plants showed lower osmotic potential, probably due to the accumulation of solutes such as proline and sugars, which helps in plant osmotic adjustment. Application of AMF to NaCl-treated plants decreases the acid and alkaline phosphatases. These results are in accordance with Beltrano et al. (2013) in pepper. The reason behind the decrease in acid and alkaline phosphatase activities may be that AMF provides P to the plant from the soil. Fujita et al. (2010) reported that activity of phosphatases in roots increases when P availability decreases in the soil.

### AMF Improved the Total Phenolics, Flavonoids, and Phytohormones in Mustard Plants under NaCl Stress

Phenolics are those secondary metabolites, which are involved in important plant functions like defence, etc. These are non-enzymatic antioxidants and are responsible for scavenging of toxic radicals (Michalak, 2006; Bartwal et al., 2013; Tomar and Agarwal, 2013) and provide membrane stability (Michalak, 2006; Khattab, 2007). Present study reported increased synthesis of phenolics in *Brassica* plants under salt stress. IncreaseS in synthesis of phenolics are also reported in *Anethum graveolens* by Mehr et al. (2012), in wheat by Tomar and Agarwal (2013) and in faba bean by Dawood et al. (2014) under salt stress conditions. Wada et al. (2014) suggested increased aggregation of phenolics in plants under stressful conditions could be attributed to enhanced activity of enzymes associated with their synthesis. The AMF-inoculated *Brassica* plants in our study showed further increase in the phenolic content. Our results corroborate with Nell et al. (2009), who has also reported enhanced phenols in *Salvia officinalis* L. inoculated with AMF. Thus, the enhanced synthesis of phenols ameliorates the negative effects of salt stress, in the presence or absence of AMF inoculation.

The article "Mitigation of NaCl Stress by Arbuscular Mycorrhizal Fungi through the Modulation of Osmolytes, Antioxidants and Secondary Metabolites in Mustard (Brassica juncea L.) Plants" was retracted in 2016. Reasons: manipulated results; errors in the data; errors in the methods; unreliable results or conclusions.

NaCl-treated plants showed enhanced accumulation of flavonoids in the present study. Similar reports are there in barley (Ali and Abbas, 2003) and *Carthamus tinctorius* (Gengmao et al., 2015). Plants accumulating higher levels of flavonoid content showed greater NaCl tolerance as compared to less flavonoid-accumulating plants (Wahid and Ghazanfar, 2006). AMF colonization further increases the flavonoid concentration in the present study. The secondary plant metabolites which lack N in their structure such as lycopene, phenolics, and flavonols are favored under conditions of reduced N. This favor continues till the photosynthetic activity is not reduced. Contrarily, N-containing compounds are favored when N is readily available to the plants (Lingua et al., 2013).

The decrease in auxin (IAA) content under NaCl stress found in the present study coincides with the finding of Nilsen and Orcutt (1996) in rice seedlings. Zörb et al. (2013) also reported decreased levels of IAA and IBA in sensitive maize cultivar. IAA decreases in roots and leaves of wheat under water deficit (Nan et al., 2002), thus hampers root growth (Egamberdieva, 2009). Exogenous application of IAA enhances root and shoot growth of wheat seedlings, suggesting that NaCl-induced decrease of root and shoot length may be due to decreased IAA concentration (Javid et al., 2011). In our study, ABA was also increased under NaCl stress and our results coincide with the findings of Zörb et al. (2013). Jia et al. (2002) also reported up to 10-fold accumulation of ABA in *Zea mays* under NaCl stress. AMF increases the IAA and IBA levels in NaCl-treated *Brassica* plants in our study, which is also reported by Luo et al. (2009). The main function of plant hormones is to participate in the AM colonization process apart from their involvement as signaling molecules (Ludwig-Müller, 2000). AMF-inoculated *Brassica* plants showed decline in ABA accumulation and the results coincide with Estrada-Luna and Davies (2003) in *Capsicum annuum* and Jahromi et al. (2008) in *Lactuca sativa* plants. Lower levels of ABA in AMF-treated plants suggested that plants are less stressed than plants under NaCl stress (Aroca et al., 2013).

The article "Mitigation of NaCl Stress by Arbuscular Mycorrhizal Fungi through the Modulation of Osmolytes, Antioxidants and Secondary Metabolites in Mustard (Brassica juncea L.) Plants" was retracted in 2016. Reasons: manipulated results; errors in the data; errors in the methods; unreliable results or conclusions.

## Conclusion

Salinity tolerance is a complex phenomenon, which is usually an amalgamation of several adaptive attributes. Increased production of ROS as a result of salinity-induced oxidative stress results in membrane damage, reduced photosynthesis, and growth retardation. Tolerance mechanisms such as enhanced activities of antioxidative enzymes, accumulation of osmolytes, increased levels of phenolics and flavonoids, among others, in response to environmental extremes are usually considered as potent defence mechanisms against salt-induced changes. The present work suggests that AMF can be helpful in counteracting the saline stress and maintaining the plant growth and development. Increase in antioxidant enzyme activities (SOD, CAT, APX, and GR), proline, phenolics and flavonoid contents, as well as reduction in H_2_O_2_ accumulation, lipid peroxidation occurring in AMF-inoculated plants justifies the key role of AMF in promoting the growth of plants under salinity stress.

## Author Contributions

MS, PA, and MA designed and performed the experimental work. PA, AH, EA_A, AA, and MA wrote the manuscript. SG carried out the statistical analysis and formatting of the paper.

## Conflict of Interest Statement

The authors declare that the research was conducted in the absence of any commercial or financial relationships that could be construed as a potential conflict of interest.
